The article "Efficacy of Sertraline Combined with Cognitive Behavioral Therapy for Adolescent Depression: A Systematic Review and Meta-Analysis" was retracted in 2023. Reasons: signs of a paper mill; compromised peer review; unreliable results or conclusions.

# Efficacy of Sertraline Combined with Cognitive Behavioral Therapy for Adolescent Depression: A Systematic Review and Meta-Analysis

**DOI:** 10.1155/2021/5309588

**Published:** 2021-12-28

**Authors:** Wenliang Liu, Gongying Li, Congjie Wang, Xiuzhen Wang, Lin Yang

**Affiliations:** Department of Psychological, Huai'an No. 3 People's Hospital, Huai'an, Jiangsu 223001, China

## Abstract

**Objective:**

The efficacy of antidepressant drugs combined with psychotherapy is controversial; hence, this meta-analysis was conducted to assess the efficacy of the combination therapy.

**Methods:**

Relevant literature was searched in PubMed, Web of Science and Embase, Chinese databases CNKI, and WanFang Data. We included the literature on the comparison of the sertraline combined with cognitive behavioral therapy (CBT) and each treatment alone for adolescent depression published in 2000-2021. Meta-analysis was performed using Stata16.0 software.

**Results:**

A total of 421 relevant articles were retrieved, and 14 studies were finally included. In comparison with the control group (sertraline), sertraline combined with CBT achieved higher response rate (OR = 5.07, 95% CI: 3.00, 8.58) and lower incidence of adverse reactions (OR = 0.43, 95% CI: 0.24, 0.75). Before treatment, there were no significant differences in depression score, anxiety score, and symptom self-rating scale score between the two groups. After treatment, depression score (SMD = −2.79, 95% CI: -3.64, -1.94), anxiety score (SMD = −1.22, 95% CI: -1.96, -0.47), and symptom self-rating scale score (SMD = −1.73, 95% CI: -3.19, -0.27) were significantly lower in the combined treatment group than in the control group.

**Conclusion:**

Although the number of comparative trials is small, this study shows that sertraline is effective for adolescent depression, but sertraline combined with CBT is more effective. The latter can significantly reduce the incidence of depressive symptoms, anxiety, and adverse reactions in patients. Therefore, this combination therapy is recommended for the clinical treatment of adolescent depression.

## 1. Introduction

Depression is a common psychiatric disorder, especially in adolescence. Depressive disorder is a comprehensive disorder with multiple features, such as depressed mood, retardation of thinking, psychomotor retardation, cognitive impairment, and somatic symptoms [1]. It has been reported that in the United States, the lifetime prevalence of depression in adolescents aged 15 to 18 years is 11%-14%; it is estimated that 20% of adolescents have major depressive disorder (MDD) at the age of 18 years, and approximately 25% are considered to have subthreshold depressive symptoms that lead to difficulties in daily functioning [2]. Additionally, approximately half of the first onset of depression in the United States occur in teenagers [3]. Among the various causes of adolescent depression, external factors are the main ones leading to psychological or neurological disorders and ultimately depression; the further development of depression into MDD is associated with interpersonal difficulties and decreased academic performance and obesity [4]. The onset of depression is usually gradual, but sometimes it can be sudden. For most patients, the course of the disease is intermittent, and the duration, number, and pattern of attacks and the number of attacks are variable [5]. The danger is that depression can induce suicidality, especially depression in childhood or adolescence; specifically, 48% of patients with early-onset depression made a suicide attempt, while 26% of adults with depression reported a suicide attempt [6]. Given the high risk of suicide in children and adolescents, it is crucial to explore effective treatment of depression for them.

The article "Efficacy of Sertraline Combined with Cognitive Behavioral Therapy for Adolescent Depression: A Systematic Review and Meta-Analysis" was retracted in 2023. Reasons: signs of a paper mill; compromised peer review; unreliable results or conclusions.

In clinical practice, the treatment of depression mainly includes pharmacotherapy and psychotherapy, and the main drugs are tricyclic antidepressants, norepinephrine and dopamine reuptake inhibitors, and selective serotonin reuptake inhibitors [7]. Sertraline is introduced to treat-related symptoms of depression, including depression accompanied by anxiety and depression with or without a history of mania. After achieving satisfactory results, continued administration of sertraline will often be continued clinically to effectively prevent the relapse of depression [8]. Most antidepressants acting on monoaminergic neurotransmission produce initial effects within the synapse, then affect intracellular signaling and second messenger pathways, and ultimately achieve remission of depression [9]. Although antidepressants can improve the mood of patients, long-term unrestrained administration causes serious side effects, such as sexual dysfunction, weight gain, nausea, and headache [10]. It has been reported that sedative antidepressants do not improve mood in depressed patients with anxiety or insomnia as well as in depressed patients with psychomotor retardation [11]. By contrast, psychotherapy is to balance out the patient's negative thinking pattern through positive care, mainly including cognitive behavioral therapy (CBT), interpersonal psychotherapy, and acceptance and commitment therapy [12]. Among them, CBT is considered to have the best clinical effect [13]. Psychotherapy requires a long treatment cycle and is expensive [13]; so, some studies have focused on the combination of pharmacotherapy and psychotherapy and have shown positive results [14, 15]. However, there is no comprehensive evaluation of the effect of sertraline combined with psychotherapy. Therefore, this study conducted a systematic review and meta-analysis of the literature published in recent years, thus assessing the therapeutic effect of sertraline combined with psychotherapy on adolescent depression and providing provide a reference for the clinical treatment of this disease.

The article "Efficacy of Sertraline Combined with Cognitive Behavioral Therapy for Adolescent Depression: A Systematic Review and Meta-Analysis" was retracted in 2023. Reasons: signs of a paper mill; compromised peer review; unreliable results or conclusions.

## 2. Materials and Methods

### 2.1. Literature Retrieval

Relevant literature was searched in PubMed, Web of Science, Embase, China National Knowledge Infrastructure, and WanFang Data, including English and Chinese literature on the treatment of depression published from 2000 to 2021. Preliminary keywords were as follows: “sertraline” AND “adolescent depression” AND “psychotherapy” OR “pharmacotherapy.”

### 2.2. Screening Criteria

Literature that met all of the following criteria were included: (1) study design: randomized controlled trial, clinical trial, and cohort study; (2) study subjects: adolescent patients diagnosed with depression; (3) intervention: treatment group was treated with sertraline combined with CBT, while the control group was given sertraline; and (4) outcome measures: response rate, incidence of adverse reactions, depression score after treatment, anxiety score after treatment, and symptom self-rating scale score after treatment. Adverse effects included headache, nausea, hyperhidrosis, dizziness, and lethargy.

Exclusion criteria were as follows: literature not related to adolescent depression; literature in which relevant data were not provided, and the data and original text could not be obtained, literature with poor quality, missing data, duplicate literature, case reports, systematic reviews, and animal experiments.

### 2.3. Data Extraction

Two investigators independently completed the literature screening and data extraction. First, according to the literature inclusion and exclusion criteria, literature that obviously did not meet the requirements was excluded. Then, the literature that may be included in the study was identified by carefully reading the titles and abstracts and by reading the full text if necessary. The corresponding materials were crosschecked to determine the literature finally included in the study. In the process of data extraction, any disagreement would be resolved through discussion by both parties or judged by a third party. The following data were extracted from the literature: first author, year of publication, study design, and main outcome measures.

### 2.4. Statistical Analysis

All statistical analyses were performed using Stata16.0 software (StataCorp LT, College Station, TX, USA). Outcome measures were expressed as standardized mean difference (SMD) and odds ratio (OR). Heterogeneity of included studies was assessed using Cochrane's *Q* test and *I*^2^ statistics. When *P* > 0.1 and *I*^2^ < 50%, a fixed-effect model was used for meta-analysis; otherwise, a random-effect model was adopted for analysis. Stability of the overall results was evaluated by sensitivity analysis. If more than 10 studies were included, publication bias was assessed by funnel plots.

The article "Efficacy of Sertraline Combined with Cognitive Behavioral Therapy for Adolescent Depression: A Systematic Review and Meta-Analysis" was retracted in 2023. Reasons: signs of a paper mill; compromised peer review; unreliable results or conclusions.

## 3. Results

### 3.1. Basic Characteristics of Included Literature

A total of 421 articles were initially retrieved, and then 344 duplicated articles were removed. Subsequently, 49 irrelevant articles were excluded by titles or abstracts. After further reading the full text, 14 irrelevant literatures with insufficient data were excluded. Finally, 14 articles were included [14–27]. See Figure 1 for the specific literature screening process and results and Table 1 for basic characteristics of included literature. And the risk of bias graph and risk of bias summary were observed in Figures 2(a) and 2(b).

### 3.2. Response Rate and Incidence of Adverse Reactions after Treatment for Depression

Eight included studies compared the response rate between the two groups [14, 16–20, 22, 23]. No marked heterogeneity was found among the included studies (*I*^2^ = 0.0%, *P* = 0.99); so, a fixed-effect model was used for meta-analysis. The result showed that the effective rate of sertraline combined with CBT for depression was significantly higher than that in the control group (OR = 5.07, 95% CI: 3.00, 8.58, Figure 3(a)).

Four included studies compared the incidence rate of adverse reactions between the two groups [15, 16, 21, 23]. No significant heterogeneity was identified among the included studies (*I*^2^ = 19.2%, *P* = 0.294); so, a fixed-effect model was employed for analysis. The results showed that combined therapy achieved a lower incidence rate of adverse reactions in comparison with the control group (OR = 0.43, 95% CI: 0.24, 0.75, Figure 3(b)).

In addition, according to the sensitivity analysis of the meta-analysis results (Figures 4(a) and 4(b)), the pooled results of the included studies did not change much and the sensitivity was low, which confirmed that the results on the response rate and the incidence of adverse reactions were robust.

### 3.3. Depression Score after Treatment for Depression

12 included studies compared depression score before and after treatment between the two groups [14–25]. A random-effects model was used for meta-analysis of depression score after treatment (*I*^2^ = 96.3%, *P* ≤ 0.001); and the result showed that after treatment, the depression score of patients treated with sertraline combined with CBT was significantly lower than that of the control group (SMD = −2.79, 95% CI: -3.64, -1.94, Figure 5).

The article "Efficacy of Sertraline Combined with Cognitive Behavioral Therapy for Adolescent Depression: A Systematic Review and Meta-Analysis" was retracted in 2023. Reasons: signs of a paper mill; compromised peer review; unreliable results or conclusions.

In addition, the funnel plot in a symmetrical manner suggested that the possibility of publication bias in the included literature was small (Figure 6). Sensitivity analysis confirmed that the pooled effect size was still of statistical significance, and the direction of the forest plot did not change significantly before and after removal of any literature (Figure 7).

### 3.4. Anxiety Score and Symptom Self-Rating Scale Score after Treatment for Depression

Five included studies compared the difference in anxiety scores after treatment between the two groups [14, 15, 22, 24, 25]. There was significant heterogeneity among the included studies in terms of depression scores after treatment (*I*^2^ = 92.2%, *P* ≤ 0.001); so, a random-effect model was adopted for meta-analysis. The result showed that the anxiety scores of patients treated with sertraline combined with CBT were significantly lower than those of the control group (SMD = −1.22, 95% CI: -1.96, -0.47, Figure 8(a)).

Six included studies compared the difference in symptom self-rating scale scores after treatment between the two groups [14, 19–21, 26, 27]. By using a random-effect model ((*I*^2^ = 98.4%, *P* ≤ 0.001), the result demonstrated that the combination therapy achieved lower symptom self-rating scale scores compared with the control group (SMD = −1.73, 95% CI: -3.19, -0.27, Figure 8(b)). Additionally, sensitivity analysis determined that the meta-analysis results were credible (Figures 9(a) and 9(b)).

## 4. Discussion

This meta-analysis mainly analyzed the efficacy of sertraline combined with CBT in the treatment of adolescent depression; the results revealed that sertraline was effective for adolescent depression, but sertraline combined with psychocognitive therapy had a better effect and could effectively reduce the incidence of depressive symptoms anxiety and adverse reactions in patients.

Numerous meta-analyses published over the past decade have clearly shown that both psychotherapy and pharmacotherapy are effective in reducing symptoms of depression [28]. In a network meta-analysis comparing the efficacy and acceptability of antidepressant drugs for MDD, 21 highly effective drugs were finally identified; however, the analysis of pooled data could not determine the individual-level effect; so, antidepressant prescription still needs clinical judgment; inevitably, long-term drug treatment caused drug resistance of patients, and the side effects of drugs cause damage to the patient's body [29]. Cognitive behavioral therapy is a long and expensive process of replacing patients' negative thinking with healthier, positive ideas [30]. It has been shown that the combination of psychotherapy and pharmacotherapy is significantly superior to each treatment alone in terms of the effective rate and functioning and QoL [31]. However, this combination therapy has also led to a decrease in the effective rate of drugs and early emergence of drug resistance in patients [32], but this report did not specifically distinguish the types of antidepressants. In this meta-analysis, the effect of sertraline combined with CBT showed better treatment effectiveness (OR = 5.07, 95% CI: 3.00, 8.58) and lower incidence of adverse reactions (OR = 0.43, 95% CI: 0.24, 0.75). However, an important limitation in the included literature is that only a few studies reported the incidence of adverse effects, which lead to insufficient analysis and weaken the credibility of the results in the comparisons.

The article "Efficacy of Sertraline Combined with Cognitive Behavioral Therapy for Adolescent Depression: A Systematic Review and Meta-Analysis" was retracted in 2023. Reasons: signs of a paper mill; compromised peer review; unreliable results or conclusions.

According to a national survey focused on cardiovascular physicians, sertraline is the most commonly used antidepressant for depression in patients with cardiovascular disease [33]. A previous trial has concluded that the use of sertraline or citalopram should be the first step in the clinical treatment of patients with MDD and coronary artery disease [34]. And in adults with mental disorders, sertraline is the most effective drug to reduce suicidal attempts in patients compared with other antidepressant drugs [35]. In this meta-analysis, sertraline could reduce the depression score, anxiety score, and symptom self-rating scale score of adolescent depression patients, but sertraline combined with CBT was more effective. There is some heterogeneity in these indicators, which may be related to the differences in method of cognitive therapy, and occupational level of psychologists [13]. Additionally, this study has other limitations. Specifically, first, many methodological complexities in the related studies on depression cause the heterogeneity of outcome measures; second, the difficulties in the definition and diagnosis of depression lead to the deviation of studies in judging the effectiveness of treatment.

## 5. Conclusion

In summary, by using meta-analysis, this study points out that sertraline is effective for adolescent depression, but sertraline combined with CBT has better efficacy and safety. The combination therapy can effectively reduce the incidence depressive symptoms, anxiety, and adverse reactions in patients. However, these conclusions still need to be verified by more high-quality studies due to the limitations in the number and quality of included studies, the heterogeneity of psychotherapy effects, and the difficulty in diagnosing depression.

The article "Efficacy of Sertraline Combined with Cognitive Behavioral Therapy for Adolescent Depression: A Systematic Review and Meta-Analysis" was retracted in 2023. Reasons: signs of a paper mill; compromised peer review; unreliable results or conclusions.

## Figures and Tables

**Figure 1:** Flow diagram of the literature screening process.

**Figure 2:** The risk of bias graph (a) and the risk of bias summary (b).

**Figure 3:** The forest plots comparing the response rate (a) and incidence of adverse reactions (b) after treatment for depression between control and treatment group. Control group, sertraline treatment; treatment group, sertraline combined with cognitive behavioral therapy.

**Figure 4:** Sensitivity analysis of response rate (a) and incidence of adverse reactions (b) after treatment for depression.

**Figure 5:** Forest plot of depression score after treatment for depression between control and treatment group. Control group, sertraline treatment; treatment group, sertraline combined with cognitive behavioral therapy.

**Figure 6:** The funnel plot assessed potential publication bias in studies evaluating the depression score.

**Figure 7:** Sensitivity analysis of depression score after treatment for depression in control (sertraline treatment) versus treatment group (sertraline combined with cognitive behavioral therapy).

**Figure 8:** The forest plot comparison of posttreatment prognosis anxiety score (a) and symptom self-rating scale score (b) between control and treatment group. Control group, sertraline treatment; treatment group, sertraline combined with cognitive behavioral therapy.

**Figure 9:** Sensitivity analysis of posttreatment prognosis anxiety score (a) and symptom self-rating scale score (b).

**Table 1:** Basic characteristics of included literature.

Study	Year	Sample time (year.month)	Cases treat/con	Age (years)		Disease (months)		Sex (male/female)		Study design	Outcome measures
				Treat group	Con group	Treat group	Con group	Treat group	Con group		
Zhou [14]	2019	2018.03-2018.12	30/30	11.53 ± 2.35	11.54 ± 2.36	8.43 ± 1.24	8.32 ± 1.23	16/14	17/13	RCT	①, ③, ④, ⑤
Zhu [15]	2012	2008.11-2011.05	66/66	15.74 ± 1.32	15.48 ± 1.29	8.88 ± 5.93	8.56 ± 6.15	35/31	38/28	RCT	②, ③, ④
Tian [16]	2020	2017.10-2019.01	40/40	13-17	14-17	2-11	2-12	20/20	23/17	RCT	①, ②, ③
Lu [17]	2020	2017.01-2019.01	50/50	15.4 ± 1.3	15.2 ± 1.4	7.9 ± 2.1	7.8 ± 2.3	31/19	29/21	RCT	①, ③
Du [18]	2018	2016.01-2017.07	82/82	15.38 ± 1.52	15.02 ± 1.46	8.68 ± 4.15	8.14 ± 3.87	37/45	34/48	RCT	①, ③
Zhu [19]	2016	2014.04-2015.06	35/35	11.78 ± 2.37	11.68 ± 3.17	8.34 ± 2.37	9.78 ± 1.45	15/20	16/19	RCT	①, ③, ⑤
Feng [20]	2021	2017.04-2019.03	31/31	13.62 ± 1.39	13.58 ± 1.27	9.55 ± 0.31	9.63 ± 0.28	NP	NP	RCT	①, ③, ⑤
Chu [21]	2020	2017.05-2019.06	20/20	14.32 ± 2.24	14.25 ± 2.36	5.07 ± 1.21	5.35 ± 1.28	10/10	13/7	RCT	②, ③, ⑤
Yang [22]	2018	2015.03-2016.05	43/43	16.8 ± 1.2	17.5 ± 1.4	3-36	3-36	22/21	23/20	RCT	①, ③, ④
Lu [23]	2020	2018.07-2020.07	45/45	14.17 ± 2.16	15.28 ± 2.09	NP	NP	29/16	28/17	RCT	①, ②, ③
Zhou [24]	2020	2017.07-2018.12	68/67	14.74 ± 2.4	14.51 ± 2.36	6.92 ± 1.46	6.85 ± 1.51	32/36	32/35	RCT	③, ④
Melvin [25]	2006	2000.07-2002.12	25/22	12-18	12-18	NP	NP	11/14	7/15	RCT	③, ④
Wagner et al. [26]	2003	2000.01-2001.06	189/187	6-17	6-17	1.5-107.6	1.1-119.3	81/108	103/84	RCT	⑤
Donnelly [27]	2006	NP	103/96	14.0 ± 1.7	14.4 ± 1.5	NP	NP	38/65	47/49	RCT	⑤

Note: Treat: treatment; Con: control; RCT: randomized controlled trial; NR: not reported; ①: effective rate; ②: adverse effects rate; ③: depression scores after treatment; ④: anxiety scores after treatment; ⑤: symptom self-rating scale scores after treatment.

The article "Efficacy of Sertraline Combined with Cognitive Behavioral Therapy for Adolescent Depression: A Systematic Review and Meta-Analysis" was retracted in 2023. Reasons: signs of a paper mill; compromised peer review; unreliable results or conclusions.

## Data Availability

The data used to support the findings of this study are available from the corresponding author (Wenliang Liu) upon request.
